The article "Increased Expression of QPRT in Breast Cancer Infers a Poor Prognosis and Is Correlated to Immunocytes Infiltration" was published in 2022. Journal: J Healthc Eng.

# Increased Expression of QPRT in Breast Cancer Infers a Poor Prognosis and Is Correlated to Immunocytes Infiltration

**DOI:** 10.1155/2022/6482878

**Published:** 2022-03-19

**Authors:** Qun Zhang, Xinwang Ding, Hongzhao Lu

**Affiliations:** ^1^School of Biological Science and Engineering, Shanxi University of Technology, Hanzhong, Shaanxi 723000, China; ^2^Wuhan Marine Machinery Plant Co, Ltd., No. 9, Wudong Road, Qingshan District, Wuhan, Hubei 430084, China

## Abstract

Breast cancer (BRCA) is a class of highly heterogeneous tumors. There is a positive correlation between the overall survival of BRCA and immune infiltration of the tumor microenvironment. QPRT is a rarely reported cancer gene, and the underlying mechanism is poorly understood. Based on TCGA data, the role that QPRT plays in BRCA is evaluated in this study. This study used GEPIA to analyze the expression of QPRT in BRCA and, based on the survival module, assessed the impact of QPRT on the survival of patients with BRCA. Furthermore, this study collected the BRCA data set from TCGA and, through utilizing logistic regression, discussed the relationship between QPRT expression and clinical information. Cox regression analysis was used to obtain clinicopathological features relating to the total survival rate of patients with TCGA. Besides, based on the “correlation” and CIBERSORT module, the relationship between cancer immune infiltration and QPRT was analyzed in GEPIA. Tumor status, pathological staging, and lymph nodes have an obvious correlation with the rise of QPRT expression according to the logistic regression univariate analysis. In this analysis, QPRT is expressed as a categorical-dependent variable (median expression value is 2.5). Furthermore, based on multivariate analysis, independent factors for favorable prognosis include negative pathological stage, increased QPRT expression, and remote metastasis. Among them, CIBERSORT analysis found that the increase in QPRT expression will increase with the growth of the level of immune infiltration of neutrophils, B cells, T cells, and mast cells. In addition, the “correlation” module using GEPIA was used to confirm. Taking all factors into consideration, the rise in QPRT expression is related to a good prognosis and a grown proportion of immune cells in BRCA, such as neutrophils, B cells, mast cells, and T cells. These results suggest that QPRT can be used to be a possible biological indicator to evaluate the immune infiltration level of BRCA and its prognosis.

## 1. Introduction

Malignant tumors formed in epithelial tissues are the most common malignant tumors and also called cancers. Cells' unnormal proliferation and differentiation, unbridled development, metastasis, and invasion are the biological features of cancer. The occurrence of cancer can be divided into three steps: the transforming growth cancer factor, cancerous promotion, and development. It is a complex process with multiple factors and multiple steps. Infection, unreasonable diet, smoking, occupational exposure, genetic factors, and environmental pollution all affect the occurrence of cancer. The malignant tumor of breast epithelial tissue is breast cancer. Most breast cancers occur in women, accounting for 99%, and the remaining extremely small probability occurs in men [1]. Breast cancer is not a fatal disease because the breast is not a decisive organ for maintaining human life. The relationship between the cells is weak and easy to fall off, however, due to the effect of breast cancer cells without normal characteristics. Along with blood or lymph, the free cancer cells are diffused to all organs after falling off come into being to transfer, which endangers lives. So far, breast cancer has been a continual killer, seriously endangering a female's mental and physical life [2]. Since the 1970s, breast cancer's occurrence has continued to increase according to the Global Cancer 2020 Statistics (GLOBOCAN2020) released by the International Agency for Research on Cancer (IARC). Breast cancer accounts for the first malignant tumor in the world, with about 2.3 million new cases in 2020, accounting for 11.7% of all new malignancies [3]. Also, based on the Ministry of Health and Disease Prevention and Control Bureau as well as the National Cancer Center in 2009, the national female breast cancer incidence rate was about 42.55/10 million people, 51.91/10 million people in urban areas, and 23.12/10million people in rural areas. There is an obvious upward trend in rural areas [4]. Breast cancer is also the most common cause of death in women under 45 [5]. This is a significant public health issue.

Genes form the basic structure and activity form of life. As all the nucleotide sequences are required to generate functional RNA or polypeptide chains, they carry all kinds of messages about blood type, pregnancy, race, and life apoptosis. They interact with the environment and create essential physiological processes such as cell division, reproduction, and protein synthesis. As a gene for protein-coding, diseases related to QPRT (Quinolinate Phosphoribosyltransferase) contain Hypertryptophanemia and Pellagra. The correlative pathways include tryptophan utilization and super pathways of water-soluble vitamins and their cofactor metabolism. The annotations of Gene Ontology (GO) associated with this type contain protein homodimerization activity and transfers activity, transferring pentyl groups [6, 7]. Previous studies have reported that QPRT enhanced breast cancer invasiveness probably through purinergic signaling and might be a potential prognostic indicator and therapeutic target in breast cancer [8–11]. Our study found that QPRT has a clear correlation with the prognosis of BRCA.

Through GEPIA and Cox regression analysis combined with data downloaded from the public domain TCGA, the correlation between QPRT and the prognosis of breast cancer was ascertained. Besides, by using cybersport, this study examined the relative percentage of various models of TIICs (tumor-filtering immune cells) in diverse tumor situations and deeply studied the correlation between TIICs and QPRT [12]. The results can be conducive to promoting the comprehension of the potential good effects of QPRT in BRCA. Also, the possible correlation and possible operational model of QPRT and tumor-immune interaction are clarified by this study. Therefore, QPRT may be a new predictor of prognosis and immune invasion in BRCA patients.

## 2. Materials and Methods

### 2.1. Data Collection

According to the published TCGA, this study collected matched clinical information and gene expression profiles. Then, this study excluded cases with deficient or lost information on partial infiltration, age, general survival time, lymph node metastasis, TNM staging, and distant metastasis. In the end, this study discussed the cases whose clinical data meet the requirements through Cox regression analysis.

### 2.2. Survival and Expression Analysis by GEPIA

An online database called -Gene Expression Profiling Interactive Analysis (GEPIA) (https://gepia.cancer-pku.cn/index.html) was applied to assess the relevance of clinicopathologic data and QPRT expression when it comes to breast cancer. GEPIA [13] is a network assistant in studying the RNA sequencing expression of 8587 regular cases and 9736 tumors from the GTEx programs and TCGA, applying a qualified processing method. GEPIA's “Survival” Sub-assembly makes it possible to assess the relevance of QPRT expression with an estimation of BRCAs. At the same time, boxplots were expressed to make the differential expression of QPRT more apparent between normal and abnormal tissues through disease states. Apart from that, trial boxplots were expressed to figure out the difference of QPRT expression in the pathological phenomenon, applying it as the variable.

### 2.3. Quantitative Real-Time PCR (RT-PCR)

Total RNA was collected from breast cancer cells, MCF-7, and MDA-kb2 from normal breast cells by using the Beijing TransGen Biotech reagent, and the RNA was reverse transcribed into a complementary DNA (cDNA). Quantitative RT-PCR was performed for validation, and the data were calculated using the 2 CT method. The GAPDH protein was used as an internal standard control for mRNA expression. The primer sequence is as follows: QPRT Forward: 5′-GGCAGCCTTTCTGATG-3′ and Reverse: 5′-GGAGCCTACTCTCTCTCCACCA-3′, GAPDH forward: 5′-CAAGGTCATCCATGACAACTTTG-3′ and reverse: 5′-GTCCACCACCCTGTTGCTGTAG-3′.

### 2.4. Assessment of Tumor-Infiltrating Immune Cells

CIBERSORT (https://cibersort.stanford.edu/), on the basis of gene expression, can assess the situations in the expression of one set of genes related to others in the group. Therefore, TIIC concentration can be accurately perceived during this time. CIBERSORT's accordant expression dynamited rising attention on heterogeneity research of cells [14, 15]. Now, our discussion estimated the proportions of 22 TIICs in BRCA through CIBERSORT and then evaluated its relevance with survival subpopulation. In a word, the information of gene expression was started through qualified noted files and transferred to CIBERSORT, with the algorithm conducting with its default signature module at 1000 arrangement. CIBERSORT gave a *P* value for deconvolution through the sampling of Monte Carlo, making behavior of confidence in the outcomes. When *P* value <0.05, it was regarded as the principle to choose that the lymphocyte may be impacted by the expression of QPRT. To explore the relevance among 22 kinds of immune cells, we made a relevant heat guiding, a graph showing relevance between every two immune cells in the trial. At the same time, the “relevance” Formula of GEPIA was applied to definite relationships between gene markers of tumor-permeating cells and expression of QPRT in depth. The gene markers covered neutrophils, markers of B cells, natural killer (NK) cells, T-helper 2 (Th2) cells, T-helper 17 (Th17) cells, and mast cells. Former researchers gave a consult for them [16–18]. The correlation module helped chart expression scatter plots of a user‐defined gene pair from a specific cancer type, with Spearman's R and programmed data meaning. *P* value <0.01 was regarded as the entrance. To explore the relevance between 22 different immune cells, we made the relevance heat map.

### 2.5. Gene Set Enrichment Analysis (GSEA)

According to the median value of QPRT mRNA expression in breast cancer, the data from the TCGA database were divided into low expression and high expression groups. According to the default weighted enrichment method, the number of random combinations was set as 1000 times, nominal *P* value (nominal *P* values, NOM P) <0.05, false discovery rate (false discovery rates, FDR) <0.25, and GSEA2.2.1 software performed gene enrichment analysis to analyze the signaling pathways in which QPRT participated.

### 2.6. Statistical Analysis

The data obtained from TCGA were all expressed by R-3.5.3. The relevance between trial features and QPRT expression was discussed by logistic regression. The analysis of COX regression was performed to confirm all survival-relevant features in the TCGA people. A *P* value lower than 0.05 was regarded as meaningful data in this research. The relevance of gene expression was gained by data meaning and Spearman's R. If the absolute value of R was over 0.1, it was thought to be related, and if not, it was defined as statistically significant.

## 3. Consequence

### 3.1. Differential Expression and Prognosis Analysis of QPRT

The results of the GEPIA database analysis showed that high expression of QPRT was significantly associated with poor overall survival (*P* < 0.05) (Figure 1(a)).  Figure 1(b) shows the relationship between QPRT expression and tumor stage, and it shows that QPRT expression increased significantly in breast cancer I, II, III, and IV tissues (*P* < 0.05). The results of the GEPIA database analysis showed that QPRT expression was significantly increased in breast cancer tissues (*P* < 0.05) compared with normal breast tissue at 3.8, while the mean expression in normal breast tissue was only 2.2 Figure (1(c)). In Figure 1(d), RT-PCR analysis of mRNA from breast cancer cells MCF-7 and normal breast cells MDA-kb2 revealed that QPRT was highly expressed in MCF-7 in breast cancer cells compared with normal breast cancer cells MDA-kb2, which is consistent with bioinformatic predictions. RT-PCR analysis of the mRNA of breast cancer cells MCF-7 and normal breast cell MDA-kb2, showed that MCF-7 is highly expressed in breast cancer cells as compared with normal breast cancer cell MDA-kb2, which is consistent with bioinformatic predictions.

### 3.2. Multivariate Analysis and Survival Results

As indicated in Figure 1, weakened expression of QPRT is relevant with unclear overall survival (Figure 1(a), *P* < 0.001) and developed the pathological phenomenon (Figure 1(b), *P* = 0.027). Apart from that, QPRT expression in tumor samples is significantly higher. As indicated in Table 1A, Univariate conclusion with Cox regression showed that some elements covering tumor status (HR = 1.229, *P* value = 0.314), pathological age (HR = 1.031, *P* value = 0.002), lymph node status (HR = 1.635, *P* value = 0.034) beside with the expression of QPRT (HR = 1.660, *P* value = 0.046) are meaningfully related with total survival. In multivariate research (Table 1B, Figure 2), the up-adjusted QPRT expression, pathological stage, and passive distant metabolism are separate prognostic elements of pleasant estimation.

### 3.3. Relation between QPRT Expression and Clinicopathologic Variables

The potential system of QPRT expression in breast cancer needs deeper research, so we discussed and associated it with specific trial aspects in terms of lung adenocarcinoma. BRCA cases with qualified trial data were discussed by R-3.5.3. As indicated in Table 2, univariate exploration by logistic regression on the basis of QPRT expression as a categorical separation showed risen expression of QPRT related meaningfully with the lymph node (N0-N1, *p* = 0.016; N2-N0, *p* = 0.060) and pathological stage (IvsII, *p* = 0.014; IvsIV, *p* = 0.102; Ivs III, *p* = 0.036, IvsII-IV, *p* = 0.000).

### 3.4. Enrichment Analyses Associated with QPRT Using GSEA

To determine the potential function of QPRT and its potential impact on breast cancer, we identified cancer features significantly associated with QPRT by GSEA, using the QORT expression data obtained from the TCGA dataset. Based on NES, FDRq, and nominal *P* values, QPRT was enriched: stress CD22-mediated BCR regulation, heme clearance from plasma, reactive antigen-activated B cell receptor BCR, reactive action of calcium mobilization, reactor-mediated MAPK activation, phospholipids in phagocytosis, reactive generation of C4 and C2 activators, reactant FCERI mobilization, and signaling binding of scavenger receptor to ligands.

### 3.5. Relevance between QPRT Expression and Tumor-Permeating Immune Cells

Former research studies indicated tumor-permeating lymphocytes as the separated prophet of the status of sentinel lymph nodes and survival on people who have cancer [19]. So, we were trying to figure out whether QPRT expression has a relationship with immune permeation in breast adenocarcinoma. Samples with the first 1/3 and the last 1/3 QPRT expression were covered into high and low expression groups, respectively. A given computer database (CIBERSORT) was applied to study gene expression of downloaded examples to deduct the part of 22 kinds of immune cells in high and low QPRT expression groups. In the last, high and low expression groups satisfied the principle of filtering. The outcomes of CIBERSORT are shown in Figure 3. The parts of 22 different types of immune cells were rendered on it. As shown in Figure 4(a), T cells CD4 record aroused, T cells follicular assistant, T cells ontrol, monocytes, macrophages M1 and eosinophils are key immune cells impacted by QPRT expression. Thereinto, T cells follicular assistant (*p* = 0.027), T cells control (*P* < 0.001), and macrophages M0(*p* = 0.002) take a higher ratio in obvious expression group rather than low expression group. In comparison, the ratio of monocytes (*p* = 0.034) is seemingly lower. Apart from that the relevant heat map (in Figure 3(b)) indicated that the ratio of other kinds of subpopulations of TIICs was impossible to relate reasonably. “Correlation” module of GEPIA assisted us to know about the connection of gene markers and QPRT expression of other kinds of immune cells that can permeate tumors, including NK cells, B cells, neutrophils, and also T cells in special functions, like Th1, Tfh, Th2, Th17, and exhausted T cells (in Table 3). The outcome indicated that QPRT expression is relevant with almost all of the genes markers of other kinds of immune cells in BRCA. CD79A of B cell showed inverse correlations with QPRT expression. This result showed us the potential regulating role of QPRT in abundance of tumor-associated B cells. The increased QPRT expression was positively correlated with its markers such as CCR7, STAT6, GATA3, and STAT3, as well as CTLA4 and IL17A. These correlations may indicate a possible mechanism by which QPRT regulates immune cell function in BRCA. The relevance was assessed with the Spearman correlation coefficient. The outcomes of markers of B cells, QPRT and neutrophils, T cells, and mast cells were likely to CIBERSORT. Therefore, what was figured out showed that QPRT might play a significant role in controlling the enrichment of neutrophils, B cells, mast cells, as well as T cells. Deeper research studies have to be done to study whether QPRT is an important element that is relevant to the immune permeation of NK cells.

## 4. Discussion

QPRT-related diseases are currently found to include Pellagra and hyperthermia [20]. Here, we found that changes in QPRT expression levels were associated with BRCA prognosis. Independent prognostic factors with a positive prognosis are reflected by the down-regulation of QPRT expression. At the same time, a decrease in QPRT expression level is closely related to clinical features such as the status of lymph nodes and tumors. Furthermore, various immune markers and levels of immune infiltration in BRCA have also been found to be related to the expression of QPRT.

Therefore, previous research suggested that QPRT may have potential effects on tumor immunity which can be used as a promising tumor biomarker [21]. In this study, we used an online database GEPIA and found a correlation between QPRT expression and prognosis in BRCA patients. Down regulations of QPRT expression are related to the positive prognosis. The distinction in tumor tissues and the expression of QPRT in BRCA normal tissues were also investigated. The TCGA data set was downloaded to further investigate the potential operational mode in cancer and the interrelation of QPRT expression. It can be seen that it is worth noting that QPRT expression is associated with BRCA levels of immune infiltration by R-3.5.3 statistical analysis in this study. CIBERSORT analysis showed that QPRT expression was closely related to the infiltration level of monocytes, macrophages, and T cells in the BRCA. Similarly, under the tumor-immune microenvironment, the relationship between gene markers and QPRT expression in different immune cells also suggests the importance of QPRT in the regulation. Using the CIBERSORT algorithm as a starting point, there is a phenomenon that compared with the high-expression group, the low expression group had a significantly higher proportion of various T cells, monocytes, and some macrophages. Furthermore, we used GEPIA “relevant” modules to confirm this finding. T cells with different functions are represented by Th1, Th2, Tfh, and Th17. To be specific, there is a positive correlation between the QPRT expression decline and their markers like LAG3, CTLA4, and STAT6. The possible mechanisms by which QPRT regulates T cell function in the BRCA are indicated by these correlations. Furthermore, a correlation between neutrophil markers and QPRT was observed. When adjusting and soliciting BRCA immune infiltrating cells, these results suggest that QPRT exerts a significant function. When studying the function of people's tumors, most research on tumor-infiltrating immune cells (TIIC) pays attention to T cells. Others describe their reaction to rates of survival and immune checkpoint suppression [11, 22, 23]. This study provides a new reference to the developing research that discerns T cells as a positive prognostic factor.

All in all, reduced QPRT expression is associated with a good prognosis. Meanwhile, changes in QPRT expression were associated with different proportions of immune cells such as monocytes, macrophages, and T cells in BRCA. Therefore, QPRT may have an important effect on immune infiltration and may be used as a biomarker for BRCA prognosis.

## Figures and Tables

**Figure 1:** GEPIA analysis of survival results and expression differences. (a) Declined expression in QPRT correlates with good results. (b) The expression of QPRT in various disease states (tumor or normal) is not the same. (c) The expression of QPRT in different pathological stages is different. (d) RT-PCR examined differences in QPRT expression between breast and normal cells in breast cancer cells.

**Figure 2:** Expression of QPRT with multivariate Cox analysis and other clinicopathological factors.

**Figure 3:** The significantly enriched signaling pathways in the high-expression phenotypes of H2AFZ in LUAD. GSEA 3.0 software. (a) Top 10 signaling pathways for GSEA enrichment. (b) Visualization of the single-gene enrichment for the QPRT. NES: normalized enrichment score.

**Figure 4:** The alteration of immune infiltration associated with QPRT. (a) The proportion of changes in the 22 immune subtypes in the QPRT high and low expression groups in the tumor samples. (b) For T cell regulation (*P* < 0.001), T cell follicular adjuvant (*p* = 0.027), and macrophage M0 (*p* = 0.002), they account for a higher proportion in the high-expression group compared with the low expression group. Monocytes account for the reduced proportion (*p* = 0.034).

**Table 1:** Cox regression analysis results. A. According to univariate Cox regression analysis, overall survival is closely related to some factors, lymph node status (HR = 1.635, *P* value = 0.034), tumor status (HR = 1.229, *P* value = 0.314), and the expression of QPRT (HR = 1.660, *P*value = 0.046). B. Independent prognostic factors with good prognosis include negative distant metastasis, QPRT expression down-regulation, and increased pathological stage.

Clinicopathologic variable	HR (95% CI)	*P* value
A stage I-II		
Age	1.031 (1.011–1.050)	0.002
T	1.229 (0.823–1.834)	0.314
N	1.635 (1.038–2.575)	0.034
QPRT	1.660 (1.008–2.735)	0.046
B stage III-IV		
Age	1.032 (1.011–1.053)	0.002
T	1.194 (0.854–1.669)	0.300
N	1.025 (0.713–1.473)	0.895
M	3.460 (1.846–6.486)	0.000
QPRT	1.804 (1.018–3.196)	0.043

**Table 2:** Logistic regression is used to analyze the relationship between clinicopathological variables and QPRT expression. There is a remarkable correlation between age, lymph node status, and pathological stage and declined QPRT expression.

Characteristics	Total (N)	Odds ratio (OR)	*P* value
Age (continuous)	858	0.776 (0.593–1.017)	0.066
Stage (I vs. II)	656	1.581 (1.099–2.274)	0.014
Stage (I vs. IV)	173	2.422 (0.838–6.997)	0.102
Stage (I vs. III)	343	1.584 (1.031–2.432)	0.036
Stage (I vs. II–IV)	858	1.597 (1.124–3.276)	0.000
N0-N1	711	1.448 (1.072–1.955)	0.016
N0-N2	515	1.543 (0.983–2.419)	0.060
Age (continuous)	858	0.776 (0.593–1.017)	0.066

**Table 3:** The relationship between gene markers of neutrophils, natural killer (NK) cells, T-helper 2 (Th2) cells, T-helper 1 (Th1) cells, T-helper 17 (Th17) cells, follicular helper T (Tfh) cells, mast cells exhausted, and T cells and QPRT expression analyzed by GEPIA “correlation” module.

Description	Gene markers	BRCA			
		Tumor		Normal	
		R	P	R	P
B cell	CD79A	0.117*∗∗*	0.000	0.561*∗∗*	1.16E−25
Natural killer cell	KIR2DL1	0.066*∗*	0.028	0.002	0.986
	KIR2DL3	0.085*∗∗*	0.005	−0.118	0.213
	KIR2DL4	0.161*∗∗*	0.000	0.107	0.261
	KIR3DL1	0.119*∗∗*	0.000	−0.068	0.476
	KIR3DL2	0.123*∗∗*	0.000	0.068	0.472
	KIR3DL3	0.049	0.104	0.063	0.506
	KIR2DS4	0.071*∗*	0.018	−0.052	0.586

Neutrophils	CCR7	0.086*∗∗*	0.004	0.4288*∗∗*	0.001
Th1	STAT4	0.052	0.081	0.162	0.087
Th2	GATA3	−0.01	0.728	0.492*∗∗*	1.21E−16
	STAT6	0.103*∗∗*	0.001	0.340*∗∗*	0.000
	STAT5A	0.052	0.084	−0.154	0.104
	IL13	0.015	0.627	0.12	0.206

Tfh	BCL6	−0.041	0.172	−0.015	0.872
Th17	STAT3	0.021	0.482	0.398*∗∗*	0.000
	IL17A	0	0.999	0.162	0.087

T cell exhaustion	CTLA4	0.152*∗∗*	0.000	0.517*∗∗*	0.001
	LAG3	0.247*∗∗*	0.000	0.382*∗∗*	0.001

Mast cells	TPSB2	0.075*∗*	0.012	0.059	0.532
	TPSAB1	−0.01	0.728	0.098	0.302
	CPA3	0.011	0.719	0.09	0.343
	MS4A2	−0.002	0.943	0.097	0.306
	HDC	−0.055	0.066	0.253*∗∗*	0.007

Tumor means correlation analysis in BRCA tumor tissue of TCGA; normal means correlation analysis in BRCA normal tissue of TCGA.

## Data Availability

The datasets used and/or analyzed during the current study are available from the corresponding author on reasonable request.
